The article "Risk Factors of Acute Radiation-Induced Lung Injury Induced by Radiotherapy for Esophageal Cancer" was retracted in 2023. Reasons: signs of a paper mill; suspected computer-generated content; unreliable results or conclusions; lack of ethics approval or compliance.

# Risk Factors of Acute Radiation-Induced Lung Injury Induced by Radiotherapy for Esophageal Cancer

**DOI:** 10.1155/2022/2416196

**Published:** 2022-07-13

**Authors:** Faen Zhang, Lihua Liao, Song Wei, Yuqing Lu

**Affiliations:** Department of Oncology, The People's Hospital of Hechi, Guangxi 547000, China

## Abstract

**Objective:**

To investigate the risk factors of acute radiation-induced lung injury (acute RILI) induced by radiotherapy for esophageal cancer.

**Methods:**

A total of 206 patients with esophageal cancer who received radiotherapy in our hospital from January 2017 to March 2020 were selected. The general data such as gender, age, and comorbidities of the patients were collected, as well as the levels of cytokines (TNF-*α*, TNF-*β*, and IL-6) in peripheral blood before radiotherapy; radiotherapy dose-related parameters were recorded during radiotherapy. Follow-up was 12 months after radiotherapy. The patients with induced acute RILI after radiotherapy were set as the observation group (*n* = 75). Patients without acute RILI after radiotherapy were set as the control group (*n* = 131). Univariate and multivariate logistic regression analysis was performed on the risk factors of acute RILI induced by radiotherapy for esophageal cancer.

**Results:**

Univariate analysis and multivariate logistic regression analysis showed that the combined diabetes, total radiation dose, combined lung disease, physical factors (V30, Dmean), and preradiotherapy cytokine (TNF-*α*, TNF-*β*, and IL-6) elevated level was an independent risk factor for radiotherapy-induced acute RILI in esophageal cancer (*P* < 0.05).

**Conclusion:**

Concomitant diabetes, total radiation dose, lung disease, physical factors (V30, Dmean), and levels of cytokines (TNF-*α*, TNF-*β*, and IL-6) before radiation therapy are risk factors for acute RILI induced by radiation therapy in esophageal cancer. The possibility of acute RILI should be comprehensively assessed according to the patient's condition, and the radiotherapy regimen should be adjusted to reduce and avoid the induction of acute radiation-induced lung injury.

## 1. Introduction

Esophageal cancer is a malignant tumor that occurs in the esophageal epithelium. Its typical manifestation is progressive aggravating dysphagia, which is one of the main malignant tumors that threaten the health of residents [1]. The incidence and mortality of esophageal cancer vary widely in different countries, and China is a country with a high incidence of esophageal cancer and one of the countries with a high mortality rate of esophageal cancer in the world [2]. There are gender, age, and regional differences in the incidence of esophageal cancer. The prevalence and mortality of esophageal cancer in men are higher than those in women, and the peak age of incidence is 45-80 years old. The incidence of esophageal cancer in rural areas is higher than that in urban areas [3]. The preferred method of treatment for early-stage esophageal cancer is surgery. Once a patient with esophageal cancer is diagnosed, surgical treatment should be performed when physical conditions permit. Combined radiotherapy and surgery can increase surgical resection rate and improve long-term survival rate [4]. However, radiation therapy easily damages the normal lung tissue within the radiation field, which in turn causes an inflammatory response in the body, resulting in acute radiation lung injury (acute RILI) [5]. Acute RILI not only affects the efficacy of radiotherapy but also reduces the quality of life of patients and even leads to death of patients. At present, the risk factors of acute RILI induced by radiotherapy for esophageal cancer have not been fully clarified, and there may be regional differences. Therefore, this study explored the risk factors of acute RILI induced by radiotherapy for esophageal cancer in Hechi City, Guangxi, and was aimed at finding an effective preventive method for acute RILI.

The article "Risk Factors of Acute Radiation-Induced Lung Injury Induced by Radiotherapy for Esophageal Cancer" was retracted in 2023. Reasons: signs of a paper mill; suspected computer-generated content; unreliable results or conclusions; lack of ethics approval or compliance.

## 2. Materials and Methods

### 2.1. General Information

A total of 206 patients with esophageal cancer who received radiotherapy at the People's Hospital of Hechi from January 2017 to March 2020 were selected. Inclusion criteria were as follows: (1) patients with complete medical records and meeting the diagnostic criteria for esophageal cancer [6]; (2) patients who completed the first radiotherapy and subsequent radiotherapy in the People's Hospital of Hechi; (3) Karnofsky performance score (KPS) ≥ 70 points and no vocal cord paralysis; and (4) computed tomography (CT) examination showed that the tumor did not invade the aorta or tracheobronchi and other adjacent tissues and organs, and there was no obvious external invasion. Exclusion criteria were as follows: (1) patients with contraindications to radiotherapy; (2) patients with major dysfunction of the heart, liver, kidney, lung, and other organs; (3) patients with distant metastasis or esophageal fistula; and (4) patients with mental disorders and uncooperative patients.

### 2.2. Research Methods

All patients were treated with a Varian Clinac CX type 4994 linear accelerator. The radiotherapy was completed by the professional radiation therapist giving the corresponding target dose according to the patient's dose prescription. Percentage of lung volume to total lung volume when both lungs received 5 Gy, 10 Gy, 20 Gy, 30 Gy, and 40 Gy irradiation (V5, V10, V20, V30, V40), average dose of bilateral lung irradiation (Dmean), and total dose of radiotherapy wait until the data was collected.

The article "Risk Factors of Acute Radiation-Induced Lung Injury Induced by Radiotherapy for Esophageal Cancer" was retracted in 2023. Reasons: signs of a paper mill; suspected computer-generated content; unreliable results or conclusions; lack of ethics approval or compliance.

The general data of the patients were collected, including age, gender, tumor location, tumor stage, smoking history, diabetes, lung disease, concurrent chemotherapy, and KPS score.

Cytokine detection: 2 mL of peripheral blood was collected from patients on an empty stomach before radiotherapy and centrifuged at 2500 r/min for 15 min. The upper serum was taken and stored at -80°C after aliquoting. The serum levels of TNF-*α*, TNF-*β*, and IL-6 were detected by enzyme-linked immunosorbent assay using a 680 automatic enzyme analyzer (BIO-RAD, USA). The testing personnel strictly follow the instructions of the kit (Shanghai Enzyme Link Biotechnology Co., Ltd.) and the instrument to perform the testing operation: TNF-*α* kit item number: ml-E12414, TNF-*β* kit item number: ml-063192, and IL-6 kit item number: ml-E12436.

The patients were followed up for 3 months after radiotherapy. The patients with acute RILI induced by radiotherapy were set as the observation group, and the patients without acute RILI after radiotherapy were set as the control group.

### 2.3. Observation Indicators

Clinical data: age, gender, tumor location, tumor stage, smoking history, diabetes, lung disease, concurrent chemotherapy, and KPS score

Physical parameters: the percentage of lung volume in the total lung volume when both lungs were irradiated with 5 Gy, 10 Gy, 20 Gy, 30 Gy, and 40 Gy (V5, V10, V20, V30, and V40), the average dose of bilateral lung irradiation (Dmean), and total radiation dose

Cytokines: TNF-*α*, TNF-*β*, and IL-6 levels in peripheral blood serum before radiotherapy

KPS scoring standard: according to the patient's health status score, 10 points are a grade, and the highest score was 100 points. A score of ≥80 was classified as a nondependent level; that is, patients can take care of themselves; 50-70 was classified as a semidependent level; that is, patient requires partial care; a score below 50 was a dependent level; that is, patient is in complete need of care

Acute RILI evaluation criteria: evaluation of acute RILI according to Common Terminology Criteria for Adverse Events 4.0 (CTCAE v4.0). Lung injury within 3 months from the first day of radiotherapy was defined as acute RILI, so all patients were followed up for 3 months after IMRT. Repeat chest CT at follow-up. According to the American Radiation Therapy Oncology Group (RTOG) acute lung injury grading scale, (1) there were occasional cough and dyspnea or there were no obvious respiratory symptoms during exertion, and only X-ray showed that pulmonary inflammatory reaction was grade 1. (2) There were persistent cough and chest tightness, and it was necessary to use narcotic cough medicine to relieve cough, which was grade 2. (3) There was severe cough and chest tightness, and the symptoms cannot be relieved by narcotic cough medicine, and intermittent oxygen inhalation or glucocorticoid treatment was required for grade 3. (4) Difficulty in breathing, insufficiency of ventilation and ventilation, and continuous oxygen inhalation or assisted ventilation were grade 4

The article "Risk Factors of Acute Radiation-Induced Lung Injury Induced by Radiotherapy for Esophageal Cancer" was retracted in 2023. Reasons: signs of a paper mill; suspected computer-generated content; unreliable results or conclusions; lack of ethics approval or compliance.

### 2.4. Data Processing

SPSS 23.0 software was used for data statistics, categorical data were expressed by number (percentage), and chi-square test was used for comparison between two groups. Continuous data were expressed as mean ± standard deviation, and *t*-test was used for comparison between two groups. The general data of the two groups were analyzed by univariate analysis, and then, the logistic regression analysis was performed to find out the risk factors of acute radiation-induced lung injury induced by radiation therapy for esophageal cancer. Statistical difference was indicated by *P* < 0.05.

## 3. Results and Discussion

### 3.1. The Occurrence of Acute RILI in Patients with Esophageal Cancer after Radiotherapy

The follow-up results showed that after radiotherapy of 206 patients with esophageal cancer in this study, a total of 75 patients developed acute RILI, of which 55 patients had grade 1, 20 had grade 2, and no grade 3 or 4 appeared. The incidence of was 36.41%. 75 patients with acute RILI were included in the observation group, and the remaining 131 patients were included in the control group.

### 3.2. Univariate Analysis of Acute RILI Induced by Radiotherapy for Esophageal Cancer

Univariate analysis showed that there were no significant differences in age, gender, tumor location, tumor stage, smoking history, concurrent chemotherapy, KPS score, V5, V10, V20, and V40 between the two groups (*P* > 0.05). There were significant differences in the levels of diabetes, total radiotherapy dose, lung disease, physical factors (V30, Dmean), and peripheral blood cytokines (TNF-*α*, TNF-*β*, and IL-6) before radiotherapy between the two groups (*P* < 0.05), as shown in Table 1.

### 3.3. Multivariate Analysis of Acute RILI Induced by Radiotherapy for Esophageal Cancer

Multivariate logistic regression analysis showed that diabetes, total radiotherapy dose, lung disease, physical factors (V30, Dmean) increased, and cytokines (TNF-*α*, TNF-*β*, and IL-6) levels before radiotherapy increased. It was an independent risk factor for acute RILI induced by radiotherapy for esophageal cancer (*P* < 0.05), as shown in Table 2.

The article "Risk Factors of Acute Radiation-Induced Lung Injury Induced by Radiotherapy for Esophageal Cancer" was retracted in 2023. Reasons: signs of a paper mill; suspected computer-generated content; unreliable results or conclusions; lack of ethics approval or compliance.

### 3.4. Discussion

Squamous cell carcinoma and adenocarcinoma are more common in esophageal cancer. According to the location of the tumor center, it can be divided into cervical esophagus cancer, upper thoracic esophageal cancer, middle thoracic esophageal cancer, and lower thoracic esophageal cancer. Middle esophageal cancer is the most common in China, followed by lower esophageal cancer [7, 8]. Symptoms of esophageal cancer are swallowing obstruction and progressive increase. From choking on swallowing and difficulty in eating hard food, it gradually developed into difficulty in eating soft food and drinking water. Its etiology is relatively complex, and it is generally believed to be related to nitrosamines, long-term smoking and drinking, and poor eating habits, and it has a certain genetic susceptibility [9, 10]. In the treatment of early esophageal cancer, surgical resection is the first consideration for resectable esophageal cancer. However, the recurrence and metastasis rate of esophageal cancer after surgery is relatively high. Combined radiotherapy and surgery can increase the surgical resection rate and improve the long-term survival rate. Therefore, radiation therapy is the main treatment for patients with advanced disease [11, 12]. The efficacy of radiation therapy depends on the radiosensitivity, and the degree of response of different tissues and organs and various tumor tissues after exposure to radiation varies [13]. The radiosensitivity of lung tissue is high, and radiotherapy of esophageal cancer is prone to cause acute RILI complications. The clinical manifestations of acute RILI are dry cough with little sputum, dysphagia, chest tightness, and chest pain and in severe cases are dyspnea, low-grade fever, pulmonary congestion, increased alveolar fibrin exudation or formation of hyaline membranes, and finally pulmonary interstitial fibrosis [14, 15]. Acute RILI greatly affects the treatment effect and long-term survival rate of esophageal cancer and reduces the quality of life of patients. Therefore, how to prevent or reduce the concurrent acute RILI during radiotherapy for esophageal cancer has become an increasingly concerned issue for oncology workers.

The results of this study showed that V30, Dmean, and total radiotherapy dose were independent risk factors for inducing acute RILI, which was consistent with the relevant literature reports [16]. It shows that the risk of acute RILI increases significantly after radiotherapy in patients with esophageal cancer with a large area of lung tissue covered by the total dose of radiotherapy, the average dose of both lungs and the large area of lung tissue covered by the radiotherapy field. Therefore, the risk of acute RILI can be reduced by improving the radiotherapy regimen and controlling the dose of radiotherapy.

The article "Risk Factors of Acute Radiation-Induced Lung Injury Induced by Radiotherapy for Esophageal Cancer" was retracted in 2023. Reasons: signs of a paper mill; suspected computer-generated content; unreliable results or conclusions; lack of ethics approval or compliance.

In terms of cytokines, the results of this study showed that increased levels of TNF-*α*, TNF-*β*, and IL-6 in peripheral blood before radiotherapy were independent risk factors for acute RILI. When the levels of TNF-*α*, TNF-*β*, and IL-6 were higher, the risk of acute RILI was also increased. TNF-*α* can initiate an inflammatory response to play an immunoregulatory role. When the level of TNF-*α* increases, the permeability of vascular endothelial cells can be enhanced, resulting in increased vascular exudation. Second, TNF-*α* has a chemotactic effect, and a variety of inflammatory cells enter the interstitial space under this effect, thereby producing an inflammatory response. In addition, TNF-*α* also has the effect of inducing the synthesis and secretion of prostaglandins, which can aggravate the inflammatory response. TNF-*β* plays an important role in cell growth, differentiation, and immune response. Studies have shown that elevated levels of TNF-beta can increase the risk of radiation-induced lung injury. IL-6 can promote lung fibroblasts to produce a large amount of acute phase proteins such as C-reactive protein, thereby exerting inflammation and immune regulation. The inflammatory state of the body can be reflected by the level of IL-6 in peripheral blood. Therefore, elevated levels of IL-6 may be closely related to radiation-induced lung injury [17].

Pulmonary disease and diabetes were the independent risk factors for radiotherapy-induced acute RILI in patients with esophageal cancer in this study (*P* < 0.05). Before radiotherapy, patients with pulmonary diseases (such as pneumonia, lung cancer, and bronchial asthma) have increased inflammatory cytokines, and the lung tissue has been damaged by chronic inflammation. At this time, the sensitivity of the lung tissue to radiation is increased, the resistance is low, and the self-repair ability is weakened. Therefore, such patients are more likely to induce radiation-induced lung injury after receiving radiation therapy [18, 19]. In order to prevent pulmonary inflammatory damage in patients, after surgical treatment, patients can be encouraged to improve lung function through abdominal breathing and other training, so as to reduce the risk of lung injury after radiotherapy. Oxygen radicals can kill cells and aggravate tissue damage by disrupting the structure and function of cell membranes. Therefore, after radiotherapy, medical staff can give patients appropriate aerosol treatment, appropriate application of antioxidants such as vitamin C, to reduce the generation of oxygen free radicals and damage to lung tissue cells. Patients with diabetes mellitus have higher blood glucose concentration and higher intravascular osmotic pressure, which may cause damage to the rupture of pulmonary microvessels, resulting in enhanced vascular permeability and increased exudation of inflammatory substances in the radiation field. This can increase the chance of lung damage. Therefore, medical staff should pay attention to the changes of blood sugar in patients with esophageal cancer in the process of treatment. In patients with diabetes, glycemic control should be administered to reduce the risk of lung injury following radiation therapy [20]. Since this study is a single-center study, the sample size collected is small, which may have a certain impact on the results and conclusions. In the future, multicenter studies and larger sample sizes are needed to identify more significant risk factors and provide preventive guidance for radiotherapy-induced acute RILI in esophageal cancer.

The article "Risk Factors of Acute Radiation-Induced Lung Injury Induced by Radiotherapy for Esophageal Cancer" was retracted in 2023. Reasons: signs of a paper mill; suspected computer-generated content; unreliable results or conclusions; lack of ethics approval or compliance.

## 4. Conclusion

Diabetes mellitus, pulmonary disease, total radiotherapy dose, elevated physical factors (V30, Dmean), and elevated levels of cytokines (TNF-*α*, TNF-*β*, and IL-6) before radiotherapy are the risks of esophageal cancer induced by radiotherapy for acute RILI factor. Before radiotherapy, the possibility of acute RILI can be comprehensively evaluated according to the patient's condition, and the radiotherapy plan can be adjusted and prepared before radiotherapy, so as to reduce and avoid the induction of acute RILI.

## Figures and Tables

**Table 1:** Univariate analysis of acute RILI induced by radiotherapy for esophageal cancer.

Factors	Observation group (*n* = 75)	Control group (*n* = 131)	*t*/*χ*^2^	*P*
Age, *n* (%)			1.272^∗^	0.259
<60years	19 (25.33)	43 (32.82)		
≥60 years	56 (74.67)	88 (67.18)		
Gender, *n* (%)			1.037^∗^	0.311
Male	41 (54.67)	62 (47.33)		
Female	34 (45.33)	69 (52.67)		
Tumor location, *n* (%)			1.345^∗^	0.510
Upper chest	16 (21.33)	21 (16.03)		
Mid chest	39 (52.00)	67 (51.15)		
Lower chest	20 (26.67)	43 (32.82)		
TNM stage, *n* (%)			1.222^∗^	0.543
I	37 (49.33)	69 (52.67)		
II-III	26 (34.67)	48 (36.64)		
IV	12 (16.00)	14 (10.69)		
Smoking history, *n* (%)			1.656^∗^	0.198
Yes	47 (62.67)	70 (53.44)		
No	28 (37.33)	61 (46.56)		
Combined diabetes, *n* (%)			11.468^∗^	0.001
Yes	51 (68.00)	57 (43.51)		
No	24 (32.00)	74 (56.49)		
Concurrent chemotherapy, *n* (%)			0.660^∗^	0.417
Yes	55 (73.33)	89 (67.94)		
No	20 (26.67)	42 (32.06)		
Total radiation dose, *n* (%)			6.249^∗^	0.012
≤60 Gy	39 (52.00)	91 (69.47)		
>60 Gy	36 (48.00)	40 (30.53)		
Combined lung disease, *n* (%)			10.013^∗^	0.002
Yes	28 (37.33)	23 (17.56)		
No	47 (62.67)	108 (82.44)		
KPS score, *n* (%)			0.424^∗^	0.515
>80 points	23 (30.67)	46 (35.11)		
≤80 points	52 (69.33)	85 (64.89)		
Physical factor				
V5 (Gy)	4421.3 ± 586.4	4586.4 ± 591.8	1.051^#^	0.110
V10 (Gy)	4337.5 ± 536.8	4295.8 ± 574.1	0.514^#^	0.608
V20 (Gy)	2513.7 ± 581.3	2431.6 ± 562.5	0.996^#^	0.321
V30 (Gy)	1124.2 ± 359.7	843.1 ± 280.4	3.496^#^	0.001
V40 (Gy)	364.6 ± 114.4	335.3 ± 110.1	0.990^#^	0.110
Dmean (Gy)	1187.4 ± 343.6	913.4 ± 286.5	3.412^#^	0.001
Cytokines				
TNF-*α* (pg/mL)	35.48 ± 11.12	21.36 ± 7.49	5.958^#^	<0.001
TNF-*β* (pg/mL)	57.24 ± 15.92	45.67 ± 13.84	3.103^#^	0.003
IL-6 (pg/mL)	11.59 ± 3.73	7.18 ± 2.01	5.888^#^	<0.001

Note: #: *t*-test; ∗: chi-square test; KPS: Karnofsky performance score.

The article "Risk Factors of Acute Radiation-Induced Lung Injury Induced by Radiotherapy for Esophageal Cancer" was retracted in 2023. Reasons: signs of a paper mill; suspected computer-generated content; unreliable results or conclusions; lack of ethics approval or compliance.

**Table 2:** Multivariate logistic regression analysis of acute RILI induced by radiotherapy for esophageal cancer.

Factors	*B*	SE	Wald	*P*	OR	95% CI
Combined diabetes	1.848	0.910	4.124	<0.001	6.345	2.026~19.877
Combined lung disease	1.281	0.632	4.112	0.004	3.600	1.178~11.000
Total radiation dose	1.399	0.752	3.464	0.012	4.050	1.306~12.557
V30 (Gy)	0.501	0.216	5.371	<0.001	1.650	1.272~4.750
Dmean (Gy)	0.453	0.196	5.362	<0.001	1.573	1.267~4.536
TNF-*α* (pg/mL)	1.564	0.931	2.822	0.003	4.778	2.159~10.782
TNF-*β* (pg/mL)	1.462	0.698	4.386	<0.001	4.315	1.134~9.641
IL-6 (pg/mL)	1.238	0.787	2.478	0.029	3.449	1.384~9.463

## Data Availability

The labeled dataset used to support the findings of this study are available from the corresponding author upon request.
